# Gene-knockdown in the honey bee mite *Varroa destructor *by a non-invasive approach: studies on a glutathione S-transferase

**DOI:** 10.1186/1756-3305-3-73

**Published:** 2010-08-16

**Authors:** Ewan M Campbell, Giles E Budge, Alan S Bowman

**Affiliations:** 1 School of Biological Sciences (Zoology), University of Aberdeen, Tillydrone Avenue, Aberdeen AB24 2TZ, UK; 2 National Bee Unit, Food and Environment Research Agency, Sand Hutton, York, YO41 1LZ, UK

## Abstract

**Background:**

The parasitic mite *Varroa destructor *is considered the major pest of the European honey bee (*Apis mellifera*) and responsible for declines in honey bee populations worldwide. Exploiting the full potential of gene sequences becoming available for *V. destructor *requires adaptation of modern molecular biology approaches to this non-model organism. Using a mu-class glutathione S-transferase (*Vd*GST-mu1) as a candidate gene we investigated the feasibility of gene knockdown in *V. destructor *by double-stranded RNA-interference (dsRNAi).

**Results:**

Intra-haemocoelic injection of dsRNA-*Vd*GST-mu1 resulted in 97% reduction in *Vd*GST-mu1 transcript levels 48 h post-injection compared to mites injected with a bolus of irrelevant dsRNA (LacZ). This gene suppression was maintained to, at least, 72 h. Total GST catalytic activity was reduced by 54% in *Vd*GST-mu1 gene knockdown mites demonstrating the knockdown was effective at the translation step as well as the transcription steps. Although near total gene knockdown was achieved by intra-haemocoelic injection, only half of such treated mites survived this traumatic method of dsRNA administration and less invasive methods were assessed. *V. destructor *immersed overnight in 0.9% NaCl solution containing dsRNA exhibited excellent reduction in *Vd*GST-mu1 transcript levels (87% compared to mites immersed in dsRNA-LacZ). Importantly, mites undergoing the immersion approach had greatly improved survival (75-80%) over 72 h, approaching that of mites not undergoing any treatment.

**Conclusions:**

Our findings on *V. destructor *are the first report of gene knockdown in any mite species and demonstrate that the small size of such organisms is not a major impediment to applying gene knockdown approaches to the study of such parasitic pests. The immersion in dsRNA solution method provides an easy, inexpensive, relatively high throughput method of gene silencing suitable for studies in *V. destructor*, other small mites and immature stages of ticks.

## Background

The European honey bee, *Apis mellifera*, is vital to the pollination of agricultural and wild plants [1]. There is widespread concern about the worldwide decline in the abundance of *A. mellifera *[2]. The ectoparasitic Varroa mite (*Varroa destructor*) is the most important pest of *A. mellifera *and plays a central role to honey bee losses [3]. *V. destructor *originally parasitized the Asian bee (*A. cerana*) where it nearly exclusively parasitized the male bees (drones), thus making little impact on the bee colony. However, in the 1950's *V. destructor *shifted to the European honey bee (*A. mellifera*) upon which it parasitizes both the drones and female bees (workers). This shift in parasitized caste is significant because the workers make up the bulk of the adult bee population within a colony [4]. *V. destructor *entered mainland Europe in the 1970's, the USA in 1987 and the UK in 1992 and subsequently has been associated with the loss of millions of colonies [3]. The mite causes damage by feeding on the haemolymph of both the developing bee within brood cells and the adult bee. Mites also transmit a variety of pathogens, most notably deformed wing virus. In terms of both the number of enterprises affected and the impact of global food production, varroasis is arguably the most serious disease of livestock in any species. Previous control of *V. destructor *by chemical treatment is increasingly ineffective due to the development of widespread resistance in mites to the limited available acaricides [5].

There is an urgent need to harness modern molecular techniques for research into the biology and, ultimately, the control of this non-model organism, *V. destructor*. RNA interference (RNAi) is a gene silencing technique that is becoming an ever more powerful tool in investigating the functional role of specific genes that may be potential targets for chemotherapeutic intervention. The RNAi mechanism involves the *in vivo *production of small interfering RNA molecules (siRNAs) from larger introduced double-stranded RNA (dsRNA). siRNA molecules target and destroy specific mRNA, silencing the target gene at the post-transcriptional stage. RNAi has been used successfully to investigate genes in a range of invertebrate species to date including gut proteins in tsetse flies [6]; moulting genes in *Tribolium castaneum *[7], aquaporins in aphids [8], a putative prostaglandin E synthase in sealice [9] and extensively in ticks (reviewed in [10]). In most cases, administration of dsRNA to the invertebrate target is achieved by intrahaemocoelic injection, though immersion in solutions containing the dsRNA has been employed for nematodes and sea lice.

In this study, we assessed the feasibility of gene knockdown in *V. destructor *using dsRNA and determined the speed and persistence of the gene knockdown effect. Additionally, we examined less invasive methods of dsRNA administration to increase ease of experimentation and improve mite survivability. The chosen target gene was a glutathione S-transferase of the mu class. GSTs were selected for study as they have been implicated in acaricide resistance in ticks [11,12] and scabies mites [13,14] and were readily amenable to activity assays to assess the effect of gene knockdown at the translational step.

## Results

### Bioinformatics and phylogeny

Of the three putative Varroa GSTs, two belonged to the mu class and the other to the kappa GST class. The largest PCR product sequenced (563 bp) was termed *Vd*GST-mu1 and the sequence deposited to EMBL [Accession No.: FR668088]. *Vd*GST-mu1 was 100% identical to the sequence (639 bp) from a pyrosequencing project on *V. destructor *from the USA (Dr. Jay Evans, pers. comm.). Alignment of the protein sequence of *Vd*GST-mu1 (213 amino acids) with other muGSTs from a variety of acari indicated that although it constituted 88% of the estimated open-reading frame, about 27 amino acids from the N-terminus were missing (Figure 1). Motifs characteristic of muGSTs were present in *Vd*GST-mu1 as well as conserved glutathione and substrate binding sites. Notably, the mu loop in *Vd*GST-mu1 was considerably different compared to other acarine muGSTs.

**Figure 1:** **Amino acid alignment of *Vd*GST-mu1 with other acarine muGSTs**. muGSTs from two mites, *Sarcoptes scabiei *type hominis [GenBank: AY825933] and *Psoroptes ovis *[GenBank: AM991140], and from two ticks *Boophilus microplus *[GenBank: AF077609] and *Rhipicephalus appendiculatus *[GenBank: AY298732] were aligned with *Vd*GST-mu1. The boxed areas represent conserved mu-class GST motifs. Putative glutathione (black highlighted "G") and substrate (black highlighted "H") binding sites are indicated. Homology across the five acarine sequences is indicated "*" = residue identity; ":" = conserved residue and "." = semi-conserved residue.

Following alignment of the mite, tick and insect sequences, but before phyogenetic trees were constructed, the sequences were truncated by approximately 27 amino acids corresponding to those missing at the N-terminus in *Vd*GST-mu1. Neighbour-joining, minimum evolution and maximum parsimony methods gave trees with similar topology and approximate bootstrap values and so only the neighbour-joining tree is presented. The acarine muGSTs clearly separated from the most similar insect GSTs (Figure 2). Within the acarine muGSTs, ticks and mites branched into different clades. Suprisingly, the *Vd*GST-mu1 did not branch with the mite clade, but rather were located in a clade containing tick muGSTs. Concordantly, *Vd*GST-mu1 shared a higher amino acid homology with ticks (e.g. *Rhipicephalus appendiculatus*, [GenBank: AY298732.1], 58% identity; *Ixodes scapularis*, [GenBank: XM_0024017051.1], 45% identity) than with mite muGSTs (e.g. *Sarcoptes scabei hominis*, [GenBank: AF462190.1], 38% identity; *Dermatphagoides pteronyssimus*, [GenBank: AY825938], 35% identity).

**Figure 2:** **Phylogeny of the acarine muGST family**. Phylogenetic tree constructed using amino acid sequences with neighbour-joining method using MEGA (4.1). Numbers are bootstrap values. Accession and database sequence identifiers are as follows: *Sarcoptes scabiei *type hominis muGST [GenBank: AY825933]; *S. scabiei *type canis muGST [GenBank: ACX33874.1]; *Lepidoglyphus destructor *allergen Lep, [GenBank: AY291572]; *Psoroptes ovis *muGST [GenBank: AM991140]; *Suidasia medanensis *Sui m 8 allergen, [GenBank: AY800356]; *Dermatophagoides pteronyssinus *muGST-2 [GenBank: AY825939]; *D. pteronyssinus *major allergen Dp15 GST homolog [GenBank: S75286]; *D. pteronyssinus *muGST-1 [GenBank: AY825938]; *Rhipicephalus appendiculatus *GST [GenBank: AY298732]; *Ixodes scapularis *GST [GenBank: XM_002401705]; *Boophilus microplus *GST [GenBank: AF077609]; *Dermacentor variabilis *[GenBank: EU551607]; *Drosophila melanogaster *GST-S1 [GenBank: NM_166217]; *Apis mellifera *GST [GenBank: FJ374871]; *Pediculus humanus corporis *GST [GenBank: XM_002426842]*; Tribolium castaneum *GST [GenBank: XM_962313]. The tree was rooted using the *S. canis *var. delta-GST [GenBank: AY649788] as the outlier.

### Tissue distribution of three *V. destructor *GSTs

RT-PCR analysis of the three cloned GSTs demonstrated marked differences in both their abundances and tissue distributions (Figure 3). *Vd*GST-mu1 seemed to be an abundantly expressed gene that was expressed at a similar level in all three dissected tissues examined, namely synganglia, Malpighian tubules and the gut. In contrast, *Vd*GST-mu2 is a less abundantly expressed gene that was clearly expressed in the synganglion and Malpighian tubules, but expressed at a much lower level in gut tissue. *Vd*GST-kap was by far the least abundantly expressed of the GSTs studied, with a slightly higher level in the Malpighian tubules than the synganglion or gut.

**Figure 3:** **Tissue specific expression of three GSTs in *V. destructor***. Expression of *VdGST *transcripts were determined by RT-PCR in different tissues of *V. destructor *using mu1, mu2 and kappa *Vd*GST-specific primers and gel loading normalized to actin. Syn = synganglion; Mal = Malpighian tubules.

### Effectiveness and persistence of *Vd*GST-mu1 knockdown in *V. destructor*

dsRNA was administered to *V. destructor *by intrahaemocoelic injection with a 20 nl bolus in distilled water and the mites then allowed to feed on bee larvae. The transcript level of *Vd*GST-mu1 was monitored by RT-PCR at various time points over the following 3 days (Figure 4). No effect was observed at 18 or 24 hr after the dsRNA injection, but by 48 hr ds*Vd*GST-mu1 injected mites had a 30-fold decrease of *Vd*GST-mu1 mRNA compared to dsLacZ injected mites (P < 0.001, Figure 4B), that represented an almost total knockdown of the target transcript and which was uniform across the three individual mites tested. By 72 h, the effect of the RNAi treatment at the transcript level was still present (P < 0.001).

**Figure 4:** **Extent and persistence of dsRNA-*Vd*GST-mu1 gene knockdown in adult *V. destructor***. (A) *Vd*GST-mu1 transcipt levels were determined by RT-PCR up to 72 h post-dsRNA treatment and gel loading normalized to actin. (B) Semi-quantitative *Vd*GST-mu1 RT-PCR band intensities were determined by densitometry and the relative abundance to the within-sample actin band calculated. The extent of *Vd*GST-mu1: actin knockdown is presented as a percentage for *Vd*GST-mu1-dsRNA injected mites and control mites injected with LacZ-dsRNA at each given time point. Data are means ± SEM (n = 3). Asterixes represent significant difference (P < 0.001) between treatments determined by Student's t-test.

### Effectiveness and mortality rates of different routes of dsRNA administration

Though microinjection of dsRNA had very effectively knocked down *Vd*GST-mu1 mRNA levels (96 ± 3.7%, n = 4, Figure 4B), such injection techniques were laborious, required specialised equipment and led to high mortality rates in the mites (50% survival, n = 62). Alternative, less invasive approaches to dsRNA administration were assessed (Table 1). A 1 μl droplet of 0.2% Triton-X100 (v/v) placed on mites immobilised on adhesive tape rapidly killed the mites (n = 6), whereas a 1 μl droplet of dsRNA in plain water had no mortality (100% survival, n = 14), but was totally ineffective in reducing *Vd*GST-mu1 transcript levels. Mites completely submerged in 0.2% Triton-X100 died very quickly (n = 15), whereas mites submerged in water died within a few hours (n = 15). Increasing the osmolality of the soaking solution by using 0.9% saline greatly increased survival of mites (72% survival, n = 26) submerged for 14 h at 4°C and then placed on bee pupae for a further 48 hr. This method effectively knocked down *Vd*GST-mu1 mRNA (87 ± 0.7%, n = 3; Figure 5). It should be noted that mites removed from brood cells and placed on bee pupae in Petri dishes but receiving no treatment at all, typically exhibited survival from 75 - 90% over a 48 hr period.

**Table 1:** Mortality of *V. destructor *and the degree of gene knockdown under different RNAi experimental conditions.

Treatment	Application Route	Survival at 48 h (%)	***Vd*GST*Mu *knockdown (%)**^**a**^
dsRNA in 0.9% NaCl	topical droplet	79 (n = 14)	0% (n = 3)
dsRNA in 0.2% Triton-X100	topical droplet	0 (n = 6)	n/d
distilled water	immersion	0 (n = 15)	n/a
0.2% Triton-X100	immersion	0 (n = 15)	n/a
0.9% NaCl	immersion	80 (n = 15)	n/a
dsRNA in 0.9% NaCl	immersion	76 (n = 21)	87 ± 0.7% (3)
dsRNA	injection	50 (n = 62)	96 ± 3.7% (4)

^a ^n/d, not determined; n/a, not appropriate; data presented mean ± SEM

**Figure 5:** **Effectiveness of gene-knockdown of *Vd*GST-mu1 in *V. destructor *following immersion in dsRNA solution**. Adult *V. destructor *were soaked overnight at 4°C in dsRNA in 0.9% NaCl. Mites (n = 3) were assayed by RT-PCR at 48 h post-treatment and gel loading normalized to actin.

### Phenotype of *Vd*GST-mu1 knockdown mites

To determine that the knockdown effect of treatment with either dsRNA-lacZ or dsRNA-*Vd*GST-mu1 was not simply just at the mRNA (transcriptional) level, but was also carried through to the protein (translational) level, we assessed total GST catalytic activity in mites (Figure 6). Mites injected with dsRNA-*Vd*GST-mu1 exhibited significantly (P < 0.05) lower GST activity rates than those injected with dsRNA-lacZ (28.1 ± 7.9 vs. 61.2 ± 12.9 FLU min^-1^).

**Figure 6:** **Total GST catalytic activity in *V. destructor *following *Vd*GST-mu1 knockdown**. GST activity of pairs of mites 48 h-post-injection with either *Vd*GST-mu1 or LacZ-dsRNA measured by monitoring fluorescence of the substrate MCB over 10 min. Closed circles represent LacZ-dsRNA injected mites (n = 4) and open circles represent *Vd*GST-mu1-dsRNA injected mites (n = 7). Data are means ± SEM.

## Discussion

GSTs are a large family of multifunctional enzymes [15] that catalyse the conjugation of reduced glutathione to the electrophilic centres of lipophilic compounds rendering them water soluble, less toxic products that can be rapidly excreted from the organism's body. As such, GSTs play an important role in phase II detoxification of both endogenous and xenobiotic compounds such as pesticides. Specifically, GSTs have been shown to be involved in acaricide resistance in ticks [11,12], scabies mites [13,14] and plant mites [16]. In the present study we demonstrated the presence and tissue expression of two mu- and one kappa-class GST in *V. destructor*. The largest sequence fragment termed, *Vd*GST-mu1 was 100% identical to the sequence present in an ongoing pyrosequencing project (Dr. Jay Evans, personal comm.) performed on *V. destructor *samples from the USA. *Vd*GST-mu1 was present in all mite tissues assessed and was, by far, the most abundant of the three GSTs examined. *Vd*GST-mu1 contained conserved glutathione and substrate binding residues and motifs characteristic of mu-class GSTs. However, both the mu-loop and SNAIL/TRAIL motifs were notably different from those of other acarine muGSTs. Interestingly, *Vd*GST-mu1 was more similar to tick muGSTs than that of mites.

*Vd*GST-mu1 was used as a test gene to assess the feasibility of dsRNAi gene knockdown in *V. destructor*. Essentially total suppression of *Vd*GST-mu1 expression was achieved within 48 h after an intrahaemocoelic bolus injection of dsRNA and this suppression was maintained until at least 72 h. RNAi by injected dsRNA is an extensively employed approach for research in ticks (reviewed in [10]) and total gene knockdown can be maintained for up to, at least, 9 days [17]. However, *V. destructor *are considerably smaller (1 mm length × 1.5 mm width) than adult ticks and injection was only possible by pulled-glass capillary needles connected to a relatively sophisticated micro-injector system, rather than using manually operated micro-syringes as is the case for ticks and most insects. Even though the micro-injector system allowed us to demonstrate effective dsRNAi in *V. destructor*, survival of mites undergoing this very invasive and traumatic procedure was only 50% over a 48 h period.

Various less invasive techniques of introducing dsRNA into *V. destructor *were investigated that would improve speed, ease of operation, increase throughput, could be performed without expensive equipment and, most importantly, increase survivability of the treated groups. Topically applied dsRNA to immobilized mites for several hours failed to induce gene knockdown, presumably because the dsRNA was unable to cross the cuticle. We tried the addition of the detergent Triton X-100 to break the surface tension of the water allowing the dsRNA solution to become more in contact with the cuticle rather than held off it by the fine hair layer (Figure 7). However, Triton X-100 caused rapid death of the mites. Next we assessed total immersion of mites as a possible route for dsRNA administration as was previously successfully performed with salmon lice in seawater [9]. Mites immersed in 0.2% Triton X-100 died rapidly and, surprisingly, mites in distilled water died within a few hours. We postulated that the hypo-osmolarity of the distilled water caused an osmotic influx of water into the mite tissues and this was exacerbated in the presence of Triton X-100 which may have allowed water to enter through the spiracles more rapidly with the reduced water tension.

**Figure 7:** **Injection sites of *V. destructor *adult female**. Arrows indicate injection sites either between the soft tissue proximal to the anal region and postcoxal plate (a), or in the soft tissue in coxal region IV (b). Scale bar = 500 μm.

Increasing the osmotic concentration of the immersion solution by using 0.9% NaCl allowed the mites to remain under solution overnight at 4°C with 75-80% survival and achieved excellent gene silencing. It is not known what is the site of dsRNA entry into the mite, but this is of considerable interest and importance. We presumed entry to be either by ingestion or though the tracheal system via the spiracles. Adult female *V. destructor *enter the prepupal cells 24 - 48 h before the cell is capped and they remain hidden from vigilant nurse bees by submerging themselves in the liquid brood food [18] with the peritremes surrounding the spiracles protruding from the liquid enabling the mites to breathe [19,20]. It may be possible to improve survivability and, possibly increase gene knockdown efficacy, if the osmolality of the immersion solution were increased to that of liquid brood food that is presumed to be greater than that of physiological saline (0.9% NaCl). Indeed, further optimisation of this approach could be attempted, if thought necessary, by altering immersion temperature and time, but the method presented here is a good starting point.

Not only was gene knockdown achieved at the transcriptional step (mRNA) but this was also apparent at the translational step (protein) with decreased GST catalytic activity. The apparent discrepancy between a 97% reduction in *Vd*GST-mu1 transcript level and the 54% reduction in GST enzyme activity is because the enzyme assay detects total GST activity not just that contributed by *Vd*GST-mu1. There have been reports of so-called "off-target" effects of RNAi whereby unintended genes sharing stretches of identical homology can be affected. A meta-analysis of dsRNAi studies in *Drosophila *high-throughput screens indicated that dsRNAs containing ≥ 19 nucleotide perfect matches to unintended targets can, in some instances, result in off-target effects [21]. In the case of *Vd*GST-mu1, the most similar gene we know of in Varroa is *Vd*GST-mu2 [EMBL Accession No.: FR675857] which shares 29% identity at the nucleotide level, but the greatest matching stretch possible is one of 12/19 nucleotides (Figure 8). Thus, it is likely that the reduction in assayable total GST activity is due to a specific knockdown of *Vd*GST-mu1, but further studies would be necessary to confirm this. Our data would indicate that *Vd*GST-mu1 is the predominant catalytic GST in *V. destructor *and highlights the specificity advantage of gene knockdown over chemical enzyme inhibitors which simultaneously affect multiple gene products.

**Figure 8:** **Alignment of *Vd*GST-mu1 and *Vd*GST-mu2 indicating stretches of perfect identity**. Nucleotide sequences of *Vd*GST-mu1 [EMBL: FR668088] and *Vd*GST-mu2 [EMBL: FR675857] were aligned using ClustalW2 and edited in JalView Vers 2.5.1 [28] with gaps not permitted and consensus stretches shown.

## Conclusions

In conclusion, we have established dsRNA knockdown in the critically important bee parasite, *V. destructor*, using a mu-class GST as the candidate gene. A simple, inexpensive, high throughput method of dsRNA administration was established with low mortality rates for *V. destructor*. This immersion approach may be applied to other small acarine pests such as scabies mites, sheep scab mites, poultry mites and plant pest mites. Additionally, the approach can be employed in ticks where the immersion approach is more convenient than injections for adult ticks but can also be applied to the smaller larval and nymphal stages which are presently not included in such gene knockdown studies. The degree of knockdown was essentially complete and persisted for several days and was apparent at both the transcript and protein level. The dsRNAi approach will allow researchers to make full use of the *V. destructor *gene sequences becoming available to investigate biological questions in this important parasite, notably to develop control strategies in the era when current suitable acaricides are no longer effective due to widespread resistance. Peculiarly to Varroa, because of the relatively close relatedness between the parasite and host (Varroa and bee) it is especially difficult to develop pesticides effective against the Varroa, but innocuous to the bee. In this respect, the specificity of dsRNAi may allow targeting of *V. destructor *genes as a control strategy, as suggested for other insect pests [22].

## Methods

### Mite collection and husbandry

*Varroa destructor *mites were collected from capped brood cells of *Apis mellifera *from hives in York, England that had purposefully been untreated for Varroa control. Prior to harvesting mites, the bee frames were maintained in Aberdeen at 27ºC and 40% relative humidity with a 15.5 h : 8.5 h, light:dark regime. Mites were either removed from newly emerged adult bees or from pupae following uncapping of the brood cell and extraction of the pupae. Mites were collected, bisected and placed in RNA ZR extraction buffer (Zymo Research, Orange, California, USA) and stored at -80 ºC prior to initial total RNA isolation.

### RT-PCR of GSTs from *V. destructor*

Six adult (pharate and mobile) and 2 deutonymph mites were homogenized in 600 μl extraction buffer and total RNA prepared using a mini RNA Isolation II Kit (Zymo Research), as per manufacturer's instructions. Eluted RNA was co-precipitated with glycogen in 95% ethanol and resuspended in 10 μl of DEPC-treated water. After isolation, 2 μg total RNA was DNase treated with 2 μl (2U) RQ1-DNase (Promega, Southampton, UK) and 2 μl RQ1 buffer and incubated at 37°C for 30 min. DNase-treated total RNA (2 μg) was incubated at 70°C with 0.5 μg of oligo d(T)15 (Promega) in a total volume of 10 μl for 5 min. Material was snap-chilled on ice for 5 min prior to the addition of 5 μl 5×RT buffer, 1 μl dNTPs (25 mM each), 0.5 μl Bioscript-reverse transcriptase and DEPC water to 25 μl. The reaction was incubated at 42°C for 60 min prior to arrest by heating to 70°C for 5 min.

A *V. destructor *database from an ongoing pyrosequencing project (Dr. Jay Evans, pers. comm.) was mined for putative *V. destructor *GST sequences by BLASTx analysis using GST sequences from the deer tick, *Ixodes scapularis*. Of 14 putative *V. destructor *GST partial sequences identified, we chose three to evaluate further: two mu-class GSTs (*Vd*GST-mu1 and *Vd*GST-mu2) and one kappa class (*Vd*GST-kap). These *Varroa *transcripts were isolated by RT-PCR using primers based on these sequences. PCR reactions consisted of 1 μl cDNA template, 5 μl 10 × reaction buffer, 2 μl 50 mM MgCl_2_, 1 μl dNTPs (25 mM each), 1 μl each primer (10 mM each), 0.5 μl (1.25 U) Taq (Bioline, London,UK) and DEPC-treated water to give a 50 μl total volume. Primer pairs used were *Vd*GST-mu-F1 (CAAGTTAAATCTTGCGTTTCC) and *Vd*GST-mu1-R1 (CTGTCCGTCTTCATGTATGC), *Vd*GST-mu2-F1 (ACGATTTATCCGTTTTGACG) and *Vd*GST-mu2-R2 (CCAACTGATGTGTCGTTCC), *Vd*GST-Kap-F1 (TACTGGTGGTCGTTTCAGG) and *Vd*GST-Kap-R1 (CTTCATAGGCCAAGAGATGC), generating products of 494, 396 and 343 bp, respectively. PCR cycling conditions were as follows: 1 cycle of 5 min at 94°C, followed by 35 cycles of 1 min at 94°C, 1 min at 53°C and 45 s at 72°C followed by a final extension time of 15 min at 72°C. Products were visualised on an agarose gel and specific bands excised and cloned into pCR4-TOPO TA vector (Invitrogen). Purified plasmids were submitted for sequencing to Eurofins MWG (Ebersberg, Germany) from flanking T7 and T3 promoter regions to confirm the original sequence data.

### Bioinformatics

The GST class of the different Varroa sequences was determined by database searches and phylogenetic analysis. For *Vd*GST-mu1, protein sequences from various acari were extracted from both non-redundant and EST databases at GenBank by tBLASTx. Additionally, the most similar GST sequences in four model insect species for which complete genomes are available were also obtained. Protein sequences were aligned in CLUSTALW2 [23]. These sequences were used to estimate phylogeny with neighbour-joining, minimum evolution and maximum parsimony methods using MEGA version 4.1 [24]. Phylogenetic trees were constructed with 10,000 bootstrap replicates.

### Expression of GST transcripts in tissues of *V. destructor*

*V. destructor *mites, were removed from brood cells, as described above, and dissected under ice-cold dissection buffer (20 mM TRIS, 5 mM EDTA, 0.9% NaCl, pH 7.4). Malpighian tubules, gut and synganglia and were dissected from 20, 25 and 98 mites respectively, washed in fresh ice-cold dissection buffer and stored in 50 μl RNA*later *(Sigma, Poole, UK) at -80 °C. Prior to RNA extraction, an additional 450 μl dissection buffer was added to sample tubes and centrifuged at 10,000 *g *for 15 min at 4°C. Supernatant was removed and tissue washed with fresh dissection buffer before a final spin at 10,000 *g *for 15 min at 4°C. Supernatant was discarded and 600 μl RNA ZR extraction buffer added to each tissue sample. Total RNA extraction, DNase treatment and reverse transcription were as described above. *Vd*GST-mu1, *Vd*GST-mu2 and *Vd*GST-kap transcripts in tissue-specific cDNA were assayed by PCR. PCR protocol and cycling conditions were carried out using the *Vd*GST-mu1, *Vd*GST-mu2 and *Vd*GST-kap primers, as described above over 30 cycles. Gel loading was normalized to *V. destructor *actin (*Vd*ActinF, CATCACCATTGGTAACGAG and *Vd*ActinR, CGATCCAGACGGAATACTT) generating a fragment of approximately 195 bp.

### Preparation of dsRNA

*Vd*GST-mu1-dsRNA was prepared using a BLOCK-iT RNAi TOPO transcription kit (Invitrogen), according to the manufacturer's instructions. LacZ-dsRNA was prepared and used as a negative control. Briefly, PCR was carried out as described above using adult female *V. destructor *cDNA in conjunction with *Vd*GST-mu1 specific primers (*Vd*GST-mu1 F1/R1), or with control LacZ-plasmid and LacZ specific primers (LacZ-F2, ACCAGAAGCGGTGCCGGAAA and LacZ-R2, CCACAGCGGTGGTTCGGAT). Products were resolved on an agarose gel, excised and purified using a Qiagen gel extraction kit (Qiagen, Crawley, UK). TOPO-T7 linker was ligated to *Vd*GST-mu1 and LacZ reactions before a secondary PCR was carried out to gain sense and antisense templates. T7-RNA polymerase was used in transcription reactions with target templates to generate sense and antisense RNA. Finally, RNA strands were annealed and the resultant dsRNA purified and quantified in a micro-spectrophotometer (Nanodrop Technology Ltd). dsRNA was ethanol precipitated and resuspended in DEPC-treated water to a working concentration of 2.5 μg/μl and stored at -80°C.

### Protocol of dsRNA injection and soaking

Adult female *V. destructor *were removed from capped brood cells along with associated bee larvae. Microinjections were carried out using pulled glass capillary needles in conjunction with a Harvard micro-injector system. Mites were placed on double-sided tape ventral side up, and injected with 20 nl (2.5 μg/μl) of either *Vd*GST-mu1-dsRNA or LacZ-dsRNA in either the soft tissue proximal to the anal region and postcoxal plate, or in the coxa IV region, as indicated in Figure 7. Needles were left in each mite for 1 - 2 min to reduce the expulsion of fluid from the wound and withdrawn slowly. Mites were left for 1 - 2 min to allow the injection site to "seal" then returned to Petri dishes containing 1 bee larvae per 4 mites. Dead or unhealthy looking mites were removed after 1 hour and mortality was monitored over 72 h in LacZ-dsRNA, *Vd*GSTmu1-dsRNA and non-injected mites.

To assess non-invasive techniques for dsRNA delivery, mites were either completely immersed in dsRNA or were exposed to a droplet of dsRNA on their ventral carapace. For soaking experiments, adult mites were removed from capped brood cells and placed in 500 μl microfuge tubes containing 20 μl *Vd*GST-mu1-dsRNA or LacZ-dsRNA (2.5 μg/μl) supplemented with either nothing, 0.9% NaCl, 0.2% Triton-X100 or both. Mites were soaked at 4ºC overnight before being removed, dried and placed in Petri dishes at 27ºC, 95% relative humidity with bee larvae. Alternatively, a sample of mites was exposed to dsRNA by attaching them to double-sided tape and placing a 1 μl drop of *Vd*GST-mu1-dsRNA or LacZ-dsRNA (2.5 μl/μg) supplemented with either nothing, 0.9% NaCl, 0.2% Triton-X100 or both on the ventral carapace. Mortality was monitored for 48 h prior to collection and validation of knockdown.

### Validation of RNAi

To validate RNAi in injected, soaked and droplet-exposed adults, the total RNA was extracted from individual mites 48 h post-treatment. In addition, persistence of the RNAi effect was measured in injected mites by harvesting at 18, 24, 48 and 72 h. Total RNA was extracted from mites using mini-RNA isolation kit II, prior to DNase-treatment and reverse transcription, as described previously. PCR was carried out using either *Vd*GST-mu1-dsRNA or LacZ-dsRNA treated sample cDNA in conjunction with primers specific for actin or *Vd*GST-mu1 using primers and cycling conditions, as described above. Products were visualized on an agarose gel normalized to actin loading. To assess persistence and approximate % knockdown, ImageJ software was used to carry out semi-quantitative densitometric analysis on gel images.

### Glutathione S-transferase activity in RNAi silenced mites

An enzymatic assay was used to assess the effect of silencing *Vd*GST-mu1 transcript on GST enzyme activity in dsRNA-treated mites. GST activity was measured by using monochlorobimane (MCB) as the substrate, as previously described for scabies mites [25] and plant mites [26], but here we adapted it for cuvettes rather than microplates. MCB forms a stable fluorescent conjugate with reduced glutathione when catalyzed with GST. Mites injected with LacZ-dsRNA or *Vd*GST-mu1-dsRNA were harvested 48 h post-treatment and frozen at -80ºC. Mites were grouped into pairs and homogenized by milling 2 × 30 s, with a single 3 mm tungsten bead in 175 μl of ice cold 0.05 M Tris buffer pH7.5 in a mechanical tissue disruptor (TissueLyser, Qiagen). After milling, samples were disrupted further in a sonicating water bath for 3 × 20 s with chilling in between bursts then centrifuged at 10,000 *g *for 5 min at 4ºC. The supernatant was retained, subjected to three freeze thaw-cycles and sonicated for a further 2 × 20 s. Samples were then centrifuged at 10,000 *g *for 5 min at 4ºC and 150 μl of supernatant from each sample used in the GST assay. Reduced glutathione was dissolved in 0.05 M Tris pH 7.5 and MCB dissolved in methanol and added to each reaction to a final concentration of 3 mM and 0.3 mM, respectively, in a total reaction volume of 200 μl. Mite homogenate and substrate were incubated at 37ºC for 10 min with fluorescence of GSH-bimane adduct measured every 2 s using a F4500 fluorimeter (Hitachi) with emission wavelength at 465 nm and excitation wavelength at 390 nm. All results presented were corrected for non-enzymatic fluorescence obtained from samples substituting 150 μl 0.05 M Tris for the mite material.

## Competing interests

The authors declare that they have no competing interests.

## Authors' contributions

EMC participated in study conception and design, performed all the experimental work and drafted the manuscript. GEB participated in study conception, facilitated sample collection and helped draft and edit the manuscript. ASB conceived and designed the study, performed sequence analysis, statistical analysis, interpretation and drafted the manuscript. All authors read and approved the final manuscript.
